RETRACTED

# Thinking and Research on Ideology Education of University Student Based on Deep Learning in Small Sample Environment

**DOI:** 10.1155/2022/7143786

**Published:** 2022-09-09

**Authors:** Lingyun Kong

**Affiliations:** School of Marxism, Qilu University of Technology (Shandong Academy of Sciences), Jinan 250353, China

## Abstract

Building an evaluation system for new media ideology education in colleges and other higher education institutions is helpful for assessing the current ideology education and encouraging high levels of information technology integration in ideology education has emerged as a key strategy for this type of education. Based on the central tenet of deep learning theory, ideology education for university students can explore educational strategies from six perspectives in order to achieve deep learning for universities. These six perspectives are opening educational channels, integrating educational contents, assisting knowledge construction, creating educational situations, problem-solving, and developing multiple evaluations. This study proposes a deep learning-based evaluation model for ideology teaching through new media in higher education institutions and colleges, applies deep learning theory to the study's research samples, and calculates the degree of association. Test samples are used to evaluate the network, and positive test outcomes are attained. The deep learning model can effectively increase the accuracy of choosing an ideological and political education approach, as evidenced by its average ideal accuracy of 92.6 percent, which is higher than that of PS-BP and DE-BP, which are 86.4 percent and 82.2 percent, respectively.

## 1. Introduction

At present, there are still some problems in ideology education for university student, such as formalization and superficiality. Most university student cannot really understand the content of education, and they are passively educated, so they cannot achieve the unity of knowledge and action. This phenomenon belongs to shallow learning in terms of learning levels. Therefore, how to promote university students' high emotion and high behavioral involvement in ideology learning, change the relationship between teaching and learning, and realize university students' deep learning are the main problems explored in this study. Ideology education can make use of many social resources with obvious educational functions [1]. For example, the historical status of economic construction around the school, typical examples and changes in residents' lives, landmark projects of social and municipal construction, existing historical and cultural monuments, advanced model figures, and various types of cultural activity venues. Teachers may neglect the real purpose of ideology education just to complete the annual teaching plan. Teachers' attitude towards the curriculum determines the way students learn ideology education. Students also enter the classroom with their bodies, but their heads are not synchronized. This is shallow learning. Human learning activity is an extremely complex system, and the study of human learning phenomenon and its essential law has always been the focus of human attention for a long time [2].

RETRACTED

Many teachers think that their task is teaching or scientific research, and they do not care about students' ideas and things outside the classroom. Some people think that student management is just a matter for full-time student management workers in schools, and they fail to regard education as their fundamental task, instead of really forming the concept of educating all the staff. They just simply take the test scores as the evaluation standard for students. When some students' grades decline, the first thing that comes to mind is the reasons of students' intelligence or learning methods, and regardless of family factors or social factors, it will also have an impact on students' learning situation [3]. For example, some students were outstanding in middle school, but after entering colleges and institution of higher learning, faced with various pressures and lack of school care, their academic performance plummeted, and they became self-abased, autistic, and even dropped out of school too early to enter the society. For a while, they could not find an ideal job and let themselves go in society. It is easy to be influenced by the bad environment in the society, and at the same time, the society and the family fail to supervise it. As you can imagine, it is inevitable to cause harm to the society, which shows that school teachers, parents of students, and all sectors of society lack communication, go their own way, and lack unity with each other [4].

Students' intrinsic motivation and cognitive needs for in-depth learning will be boosted when the learning subject discovers that the learning object exists in the complicated problem domain of flawed structure and the genuine social context and has a moderate cognitive load. Ideology education can use a variety of instructional resources, including media, to prepare college students for a range of real-world scenarios. The inner drive for learning will be sparked when the situation conflicts with the preexisting cognition [5]. In contrast to the conventional classroom of ideological and political education, where professors and students are exclusively involved in teaching and listening, deep learning places emphasis on the development of thinking. The active classroom is important to deep learning, which also makes efficient use of time constraints. Even a dry course on ideology theory will be endlessly entertaining in such a learning environment. It can also enhance the effectiveness and quality of the ideology course's instruction at the same time. Drawing conclusions from others is valued in deep learning [6]. The fundamental goal of ideology education cannot be attained if pupils are forced to merely copy, mechanically recall information, and understand concepts at a surface level. In order for students to properly comprehend the meaning and significance of an ideology theory during the question-answering process, it is required to reinvent the teaching methods, increase the quantity of classroom questions, and innovate the questioning methods of the ideology theory course.

RETRACTED

The chapter arrangement of this paper is as follows: the first section of this paper introduces the related research of relevant scholars in the field of ideology education, the second section establishes the evaluation index of ideology education based on deep learning, the third section brings the evaluation index into deep learning model to analyze the accuracy rate of the optimal teaching strategy experiment selection strategy, and the fourth section is the full text summary.

This paper's innovation is as follows: this paper builds an evaluation model using the BPNN combination evaluation method on the foundation of a thorough analysis of several contemporary comprehensive evaluation methods. The large amount of computation required by the grey relational analysis method for evaluators is compensated for by the intelligent programming of this method, which significantly increases evaluation efficiency and makes the evaluation model more accessible to the general public.

## 2. Related Work

The rise of quality education in institution of higher learning is the requirement of social and technological development for higher education. Due to the strong impact of science, technology, and economic development, university education focuses on cultivating technical talents to adapt to economic development, and neglecting humanistic quality education has become a common problem in university education all over the world. The consensus reached through reflection on this issue is to improve the overall quality of the educated [7].

Guan thinks that the teacher holds the key to a class's quality. In the end, teaching activities are bilateral interactions between teachers and students, and the effort put forth by the students in the lead role ultimately depends on the effort put forth by the teachers. Teachers must stand at their commanding heights if they want to fully embody their leadership role and turn the restricted classroom time and space into limitless teaching time and space. One of the main responsibilities of teachers in the classroom when teaching courses in ideology is to assist students in organising their knowledge, highlighting the important ideas, and overcoming obstacles in accordance with the demands of the learning and teaching objectives, which helps students remember, apply, and remember information more easily [8]. Peng thinks from the perspective of ideology education. Intelligent algorithm brings transformation opportunities for ideology education, but it also has many negative effects. It is necessary to effectively judge the algorithm risks of ideology education, provide ideology education wisdom for optimizing and controlling algorithms, and make the algorithm technology better serve human society [9]. Ou believes that negative incentives should be used with caution for counselors engaged in student work, because punishment will bring psychological trauma to people. For our students, the negative incentives are roughly criticism, cancellation of evaluation, warning, probation, and so on. These negative incentives may serve as an example, but we must grasp the scale and strength of negative incentives and not produce any deviation [10]. Ding and Dan think that the network has the characteristics of fast operation, synchronization, and ease of use, which makes university student get information very quickly. The network supported by computer, communication, and information technology will become the link of the future information society, and it will unite all countries and regions in the world to form a brand-new information and communication network system, which can transmit and process an increasing amount of data, information, and knowledge at a faster speed. Influenced by its characteristics, university student will inevitably form a strong concept of efficiency when using the network [11]. Xuan and University think that with the deepening of global integration and economic globalization, the development of Internet technology, and the influx of various values and cultural tides are constantly impacting university students' thoughts, and some decadent lifestyles are eroding university students' minds, resulting in great changes in some university students' way of thinking [12]. Dan believes that the ideology education system is the organizational system and leadership system of ideology education in colleges and institution of higher learning, which mainly solves the problem of who should be responsible and who should manage the ideology work in colleges and institution of higher learning. At the same time, it is necessary to give full play to the role of administrative leaders, trade unions, the Communist Youth League, student unions, and other mass organizations, and jointly do a good job in ideology work [13]. According to Zhang, negative motivation is passive motivation that weakens certain human behaviours by denying, stopping, and punishing them, and by moving those behaviours in a direction that promotes the satisfaction of both individual needs and organisational objectives. Because the incentive effects of these two ways will not only directly affect individuals but also indirectly affect the surrounding individuals and groups, both positive and negative incentives are required and effective [14]. According to Liu, some university students are dislocated and inclined in concept and morality under the influence and impact of various negative factors in society, which causes the young students' thoughts to also change [15]. This is because there are still some gaps in the management of higher education. According to Xie and Lin-Hua, in the process of managing students, students are to be influenced through professional and psychological counseling so as to achieve the guiding function. In fact, it performs the function of ideology education [16]. Liu integrates ideology education into various specific student works, such as carrying out effective dormitory management and organizing students to participate in social practice activities, etc., and places ideology education in service and management [17]. Min and Marxism regard dormitory as the position of ideology education, equipped with special service personnel and tutors in dormitory area, equipped with special student accommodation assistants and consultation centers, and actively helped students to carry out various activities in dormitory, thus exerting a subtle influence on students' ideology education. Using the method of nonideology education, transmitting the essential ideology education content, such as professional team, scientific structure, good service, etc., all these show that the implementation of its ideology education has been carefully designed and organized [18].

RETRACTED

The largest flaw is that college administrators do not adequately and effectively incorporate political and ideological education into their management. As a result, the main challenge facing personnel training at the moment is how to combine ideological and political education with student management in colleges and universities. This essay investigates the methods of deep learning-based ideological and political education. Deep learning's basic function, which might be considered its main characteristic, is the development of higher-order cognitive skills. In addition to helping to realise and promote deep learning, deep learning also helps to enhance the quality of learners' thinking and the effectiveness of their learning.

## 3. Algorithm Design of Evaluation Index of Ideology Education in Colleges and Institution of Higher Learning Based on Deep Learning

### 3.1. Evaluation Model Based on BPNN Algorithm

The BPNN is a sophisticated network system that does nonlinear conversion and parallel information processing, simulating how the human brain nerve processes information [19].  Figure 1 depicts its structure.

Input layer, hidden layer, and output layer are the three or more layers of neurons that make up a BP network. The concealed layer among them might have one or more layers, and the quantity of neurons in each layer is often decided by the actual issues. Although the neurons in the same layer are not connected, the upper and lower layers are completely interconnected. The introduction of BPNN allows the evaluation model as a whole to not only compare multiple samples and the multiple factors present in each sample horizontally but also to adjust intelligently from output to input in reverse, greatly reducing the influence of human factors on the evaluation process. In addition, this method's clever programming allows computers to perform several computations simultaneously, making up for the drawback of requiring evaluators to perform a lot of calculations and significantly enhancing assessment efficiency. The ideology teaching of new media in colleges and other higher education institutions exhibits clear characteristics from the standpoint of evaluation. The ideological teaching of new media in colleges and other higher education institutions is a multifactor system, based on the composition of the evaluation object.

The ideology education system of new media at colleges and institutions of higher learning contains a lot of hazy information as far as information acquisition is concerned. In colleges and other higher education institutions, the ideology education of new media includes both direct, explicit, and immediate information that people may easily get and indirect, implicit, and long-term information that is frequently challenging to identify. A typical multifactor complex system, new media ideological and political education at colleges and universities, is particularly expressed in the educational objects, educational environment, and educational process. The algorithm acts as a go-between for people and information, and it can covertly carry out the ideology education function of influencing the audience's political preferences and ideological values. The efficacy of ideology instruction in a network setting will directly depend on how rational and successful the algorithm technology is. Determine the data sequence that can be referenced to in order to create the evaluation index. The reference data column is shown in

(1) $$\begin{array}{c} z_{0}\left(x\right)=\left\{z_{0}\left(1\right),z_{0}\left(2\right),\cdots ,z_{0}\left(c\right)\right\},x=\left(1,2,\cdots ,n\right). \end{array}$$

The compared sequence in BPNN is recorded as the subfactor time sequence, as shown in

(2) $$\begin{array}{c} \xi \left(x\right)=\frac{\underset{i}{\min}\left|z_{0}\left(x\right)-z_{i}\left(x\right)\right|+\underset{k}{\max}\left|z_{0}\left(x\right)-z_{i}\left(x\right)\right|}{\left|z_{0}\left(x\right)-z_{i}\left(x\right)\right|}. \end{array}$$

The only information provided by BPNN is the level of correlation between the data at any given time. The information is overly dispersed and makes comparisons difficult due to the high number of correlation coefficients. As a result, the correlation coefficients at each instant must be combined into a single value. One approach for handling this type of information centrally is averaging. In this example, the minimum absolute difference and the greatest absolute difference are compared.

(3) $$\begin{array}{c} \xi \left(x\right)=\frac{\Delta \underset{i}{\min}+\underset{k}{\Delta \max}\left|z_{0}\left(x\right)-z_{i}\left(x\right)\right|}{\left|z_{i}\left(x\right)-zk\left(x\right)\right|+\text{l}\Delta max}. \end{array}$$

The training sample of BPNN is shown in

(4) $$\begin{array}{c} x_{ml}=\left\{\begin{array}{ccc} x_{11} & \cdots & x_{1w}\\ x_{21} & \cdots & x_{2w}\\ \cdots & \; & \;\\ x_{q1} & \cdots & x_{qw} \end{array}\right\}. \end{array}$$

The random number is used to initialize the data, and the initial values are assigned to the connection weights and neuron node offsets of the neural network. Learning is a process of error back propagation and correction. The total error function of actual output and expected output of sample mode is shown in

(5) $$\begin{array}{c} \omega_{s}\left(x+1\right)=\omega_{s}\left(x\right)+℘nx. \end{array}$$

The algorithm is endowed with value rationality by the ideological and political education. Intelligent algorithm does not pay attention to mining the social value and lofty meaning of information, but only obeys the capital logic, thus causing some negative effects, which makes people begin to reflect on ethical issues. Ideological and political education is closely related to the algorithm, so if the algorithm wants to find the correct development direction, it must be guided by ideological and political education first. In order to evaluate the quality or grade of different ideology education strategies, a secondary index is set under the index of effectiveness of educational process, as shown in Table 1.

RETRACTED

The key to the success of creating teaching situation lies in whether it can cater to students' psychology. The content of the situation should be novel, difficult, and targeted, and should not be copied mechanically in order to create the situation, nor should it be a situation that students cannot understand, otherwise students will lose interest in learning. The process of students' self-evaluation is the process of promoting students' self-reflection. Through self-evaluation, they can clearly understand their own cognitive situation and existing problems, and develop their own metacognitive ability, which is conducive to improving their follow-up behaviours. Peer evaluation can learn from each other's strong points, correct each other, coordinate interpersonal relationships, and make common progress. Participation from the family and community in evaluation can keep up with social, academic, and family education, allowing kids to develop long-lasting, morally upright habits [20]. The extreme value normalisation method is used to standardise the index value in order to reduce the impact of each index dimension on the evaluation result and to unify the variation range of each index value. The positive index is shown in the calculation.

(6) $$\begin{array}{c} x_{ij}^{z}=\frac{x_{z}-\min\left(x_{i}\right)}{\max\left(x_{j}\right)-\min\left(x_{i}\right)}. \end{array}$$

The reverse index is shown in

(7) $$\begin{array}{c} x_{ij}^{z}=\frac{x_{z}-\min\left(x_{i}\right)}{\max\left(x_{j}\right)-\min\left(x_{i}\right)}. \end{array}$$

The objective function is defined as the product of the distance between classes of projection values and the density within classes, as shown in

(8) $$\begin{array}{c} z\left(i\right)=\overset{x}{\underset{i=1}{\sum }}a_{z}x_{ik}^{x}. \end{array}$$

Find the best projection direction by maximizing the product of the distance between classes and the density within classes, that is, find the maximum of the projection index function, as shown in

(9) $$\begin{array}{c} Z_{i}=\sqrt{\frac{\sum_{i-1}^{n}{\left(z\left(i\right)-Z\left(x\right)\right)}^{2}}{n+1}}. \end{array}$$

Read the ideology education strategy's evaluation index data, divide the training and test sets, and normalise them to remove the impact of data dimension differences. Then, determine the algorithm's termination conditions, and if the maximum number of iterations is reached, output the best solution by determining the best projection direction. For the purpose of determining the quality or grade of an ideology education approach, the optimum projection direction is entered into BPNN.

RETRACTED

### 3.2. Visualization Processing of Statistical Data

After defining the object of ideology work, ideology workers should choose appropriate time, appropriate ways, and appropriate methods to collect the ideological information of the object. According to the collected information, ideology workers can analyze the collected information according to certain methods and generate analysis results. Various models are put forward in different fields of information processing, with the aim of establishing a unified theoretical foundation for system development, application development, and education and training. Similarly, the visualization system also needs a reference model to solve related problems. Visualization is essentially a part of computer-aided postdata processing in the process of scientific research, and its purpose is to provide people with a visual analysis method. Usually, when studying a physical phenomenon, a physical model is first established, and then it is converted into a mathematical model. Based on this, the computer model is put forward and sent to the computer for calculation. The simulation result data is converted into visual graphic information for analysis and research, the correctness of the physical model is verified, and the inherent laws of the physical phenomenon are summarized. The function of data preprocessing is to standardize the original data generated by simulation to form applicable data, and then the mapping module maps it to geometric data, such as points, line segments, and polygons. Drawing is to convert geometric data into images [21].

Two-dimensional scalar field can be regarded as data distribution on two-dimensional planar grid points or scattered points, and the key is how to construct its interpolation function or approximation function. For grid data, the simplest method is to use bilinear interpolation, and only rely on four grid points to construct its interpolation function, as shown in

(10) $$\begin{array}{c} F\left(x,y\right)=\overset{2}{\underset{i=1}{\sum }}\overset{3}{\underset{i=1}{\sum }}\partial_{j}x^{i}y_{i}. \end{array}$$

Intelligent algorithm technology and tools provide innovative application services for ideology education in terms of scene reconstruction, data tracking, and resource matching, which not only promotes ideology education to be in an unprecedented open state but also constructs fragmented ideology education materials in a very flexible way, associates and integrates them into their daily online life fields, and naturally integrates life entertainment, value guidance, and knowledge education, which reflects its value function of collaborative education of ideology courses, and promotes multiagent education by following the ideology work system, as shown in Figure 2.

RETRACTED

With the difference of original data, a common visualization system may omit the data preprocessing module, or combine some data preprocessing module functions with the mapping module functions. Aiming at the problem of insufficient supply of ideology education content caused by the algorithm technology, ideology educators should make good use of the intelligent algorithm technology and actively integrate ideology education content into the algorithm recommendation pool. It is particularly important to emphasize cooperative learning among different subjects in the process of ideology education. This kind of collaboration is not only the collaboration between teachers and students but also the self-collaboration between students and students. For some topics that can be discussed, teachers can organize students to exchange and discuss, establish a common learning group, and let each student play a role and become one of them. Deep learning attaches importance to learners' transfer and application of knowledge, and requires students to not only understand the learning content but also deeply understand the learning situation. Students need to master many key elements in learning situations and make clear the differences in each situation. Therefore, in ideological and political education, we should also pay attention to the setting of learning situations and create diverse learning environments close to social reality.

## 4. Strategic Choice of Ideology Education Based on Deep Learning Model

### 4.1. Simplicity and Division of Index System

Education must start with solving the contradiction between teachers and students, and make them become teachers and students by adjusting the contradiction between both sides. Ideology courses in colleges and institution of higher learning should reexamine and construct the relationship between teachers and students, establish a student-centered teaching concept, guide students to study, explore, and create independently, explore and reflect on new knowledge, and thus construct their own knowledge system. In the teaching process, teachers of ideology courses should integrate theory with practice, seize the social hot issues that students are interested in, create a real learning situation that fits students' reality, cultivate students' interest in learning, arouse students' enthusiasm for learning, and make students explore and practice independently in active participation, so that knowledge can be understood and absorbed by students imperceptibly. Ideological and political educators can apply deep learning as a new teaching method to the ideological and political theory course, explore the operation mechanism of deep learning, and put forward some operable suggestions for the smooth development of ideological and political education, which is undoubtedly of great significance. Generally, there is no uniform measurement standard among the various characteristic indexes of the evaluated object. In order to eliminate the dimensions of the collected original data, the original data is processed by averaging to make it dimensionless. Averaging is to divide all the data by the serial average.

RETRACTED

According to the evaluation index system of ideology education, the input sample is a 50-dimensional input vector, so there are 50 neurons and 50 input nodes in the input layer. The evaluation of new media ideology education in colleges and institution of higher learning by output level is a process from qualitative to quantitative and then to qualitative. Through BP network model, the qualitative is transformed into quantitative output, and then the collective output results are comprehensively evaluated to make a qualitative evaluation of new media ideology education. Set the number of neurons in the output layer to 1. Evaluation set is the key to the whole evaluation process, and its setting will affect the objectivity of evaluation. The selection of the number of neurons is related to the accuracy and learning efficiency of the whole BP network. Therefore, when selecting the number of hidden layer energy neurons, both the accuracy of the BP network and the learning efficiency of the network should be taken into account. After many times of parameter debugging and statistical observation one by one, the number of hidden layers is finally determined to be 20. The BPNN is trained and simulated by MATLAB 8.0, and the results are shown in Figures 3 and 4.

The Figure 4 shows that the actual output and expected output are very nearly identical, and the difference between the two is within the desired range, which actively encourage the platform cooperation and intelligent transformation of information dissemination topics in ideological education. On the one hand, it is important to use the algorithms to improve the mainstream media's knowledge. The mainstream media serves as the primary channel for disseminating the informational materials used in ideology education, but there have always been problems, such as page columns that become static and information that is out of date. In order to enhance the operation of mainstream media and boost attention, page visits, and user stickiness of mainstream media, update and dynamically present the platform interface in real-time, increase the push information supply, and optimise user browsing experiences. The mainstream media, on the other hand, needs to integrate with the market-oriented media platform, create ideology education propaganda boards and link portals, rely on the technical advantages of commercial media to increase their influence, and increase the ability of positive energy information to influence online public opinion. Teachers support knowledge meaning construction in the deep learning classroom by helping students understand and adapt to the dynamic learning environment. Students take the initiative to study and even have the freedom to choose the course material. Instead of only being passive recipients of knowledge, they create the meaning of knowledge. In a deep learning setting, both teachers' and students' excitement and initiative can be mobilised simultaneously.

RETRACTED

### 4.2. Ideology Education Strategy Rating Scheme

In the teaching process, teachers of ideology courses should integrate theory with practice, seize the social hot issues that students are interested in, create a real learning situation that fits students' reality, cultivate students' interest in learning, arouse students' enthusiasm for learning, and make students explore and practice independently in active participation, so that knowledge can be understood and absorbed by students imperceptibly. Political teachers should actively create a learning environment conducive to communication, consultation, cooperation and mutual assistance, and guide students to establish different types of learning communities. Students have different understandings of things because of their own knowledge and experience, emotional attitudes, surrounding communities and cultural backgrounds, and there are individual differences in the process and results of meaning construction. Let students master the right to speak in class and put forward their own views and opinions on the key issues. Teachers do not completely retreat behind the scenes, but thread the needle in the process of students' discussion and communication, and give timely guidance, inspiration, and summary. It is particularly important to emphasize cooperative learning among different subjects in the process of ideology education. This kind of collaboration is not only the collaboration between teachers and students but also the self-collaboration between students and students. For some topics that can be discussed, teachers can organize students to exchange and discuss, establish a common learning group, and let each student play a role and become one of them. The content of collaboration includes not only the collation and induction of learning materials but also the control of learning progress and evaluation of learning results. Collaboration should run through the whole learning process. University students' classroom collaboration includes group study and discussion study, and after-class collaboration includes group investigation and student association. Students' self-cooperation is also very important, that is, judging something according to their own knowledge and experience, arguing with themselves, and exploring independently.

RETRACTED

In order to evaluate the quality or grade of different ideology education strategies, this paper selects five grades of ideology education strategies as the research object, as shown in Table 2.

In order to prove the superiority of the deep learning model in the strategic choice of ideology education, the deep learning model is compared with PS-BP and DE-BP. In the evaluation of ideology education strategy selection, different indicators are used as the input values of data, and the model of ideology education strategy selection is established. The results are shown in Figure 5.

The Figure 6 illustrates how the deep learning model can effectively increase the accuracy of ideology education strategy selection. The average optimal accuracy of the deep learning model is 92.6 percent, while the average optimal accuracy of PS-BP and DE-BP are 86.4 percent and 82.2 percent, respectively.  Figure 7 displays the results of comparing the convergence speed of the deep learning model with the PS-BP model and the DE-BP model.

The Figure 7 shows the deep learning model. It has faster convergence speed and higher evaluation accuracy. Ideology educators should use artificial intelligence technology to analyze and interpret. The birth and application of any technology means the emergence of a new evaluation scale. The algorithm technology based on utility rules aims to promote the ideology education's self-awareness, self-positioning, and self-empowerment in the network with the help of digital media, and at the same time self-adjustment, self-improvement, and self-regulation in the network survival. On the one hand, the algorithm utility rule is used to grasp the “degree” of network ideology education, and the evaluation scheme is presented and operated in the form of network platform, realizing the functions of multiport operation, multiagent participation, real-time data processing, scientific statistical analysis, and so on, so as to evaluate the level of network ideology education. Including the accuracy of specific publicity and education audience range, the height of content, the depth of analysis, the strictness of logic, and the density of education, we should also grasp the scale of ideology education, grasp the discretion, and avoid its disorientation and anomie. On the other hand, the intervention and warning based on utility rules should be set up, and the mainstream ideology and algorithm code should be related to realize the organic balance between value orientation and technological development.

RETRACTED

On the premise of ensuring personal privacy, through comprehensive collection and in-depth analysis of network data, we should establish a group social emotional risk analysis and early warning mechanism. The core goal of the system is not only to deal with the hot events on the Internet but also to accurately grasp the whole social thoughts and emotions in the future and make advance predictions, so as to minimize the destructiveness of people's stress behaviours caused by group social emotions and promote social harmony and stability. Intelligent algorithm technology can empower network ideology education to bring media, forums, Weibo, WeChat, and other channels into the scope of monitoring. With its analysis and mining ability, it can extensively investigate people's feelings and opinions, collect problem clues, comprehensively present key and emerging information about people's thoughts and emotions, and generate daily intelligent reports in real time. Intelligent algorithm analysis technology can set red-line sensitive words and alarm mechanism. When the emotional and ideological indicators of a hot event in the network exceed the safe area, it deconstructs the event according to crowd attributes, event tracking, region, and other dimensions and outputs an analysis report. Combined with human intervention decision-making, it can respond to the crisis, actively communicate, and positively guide the thoughts.

## 5. Conclusions

Nowadays, the innovation and development of ideology education must be linked with the algorithms, and the algorithms should be reflected and integrated. This integration is not simply added, but the two are embedded, infiltrated and integrated with each other. Ideology education itself mainly depends on the advantages of the algorithms to adjust the content structure and implementation logic and plays the role of guiding ideas, guarding mainstream values, and condensing social consensus. On the premise of ensuring personal privacy, through comprehensive collection and in-depth analysis of network data, we should establish a group social emotional risk analysis and early warning mechanism. The core goal of the system is not only to deal with the hot events on the Internet but also to accurately grasp the whole social thoughts and emotions in the future and make advance predictions, so as to minimize the destructiveness of people's stress behaviours caused by group social emotions and promote social harmony and stability. Intelligent algorithm technology can widely investigate people's feelings and opinions, collect clues of problems, comprehensively present key and emerging information of people's thoughts and emotions, and generate daily intelligent reports in real time. Intelligent algorithm analysis technology can set red-line sensitive words and alarm mechanism. When the emotional and ideological indicators of a hot event in the network exceed the safe area, it deconstructs the event according to crowd attributes, event tracking, region, and other dimensions and outputs an analysis report. Combined with human intervention decision-making, it can respond to the crisis, actively communicate and positively guide the thoughts. As there are many factors to choose ideological and political education strategies, this paper only considers some evaluation factors, and will study the choice of ideological and political strategies with more influencing factors in the later period to further improve the applicability and accuracy of the model.

RETRACTED

## Figures and Tables

**Figure 1:** BPNN structure.

**Figure 2:** Data visualization process.

**Figure 3:** BPNN training curve.

**Figure 4:** Actual output and expected output.

**Figure 5:** Training set.

**Figure 6:** Test set.

**Figure 7:** Comparison of convergence speed.

**Table 1:** Evaluation index of ideology education.

Primary index	Secondary index
Moral trait	Spirit of dedication
	Self-discipline spirit
	Abide by the norms of social and public life
	A healthy lifestyle
	Moral responsibility
Political behaviour or record	Ability to recognize major historical issues and judge right and wrong
	Care about national politics
	Participate in social welfare activities
	Is there a blood donation record
Ideology theory	Master of laws and regulations
	Score of ideological and moral cultivation course
	Mastery of modern Chinese history
	With the situation and policy to understand the situation with politic
Daily performance	Attitude towards participation in class public activities
	Classroom order compliance
	Good living habits
	And personal hygiene in gfd.
	Help students who live actively and think backward
Learning index	Borrowing amount
	Time in the library

**Table 2:** Grade evaluation of ideology education strategy.

Grade	C1	C2	C3	C4	C5	C6	C7
Excellent	>100	>1	>20	>20	>500	90~100	80~100
Better	80~100	0.5~1.0	10~20	10~20	100~500	80~90	50~80
Middle	60~80	0.1~0.5	5~10	5~10	50~100	50~80	10~50
Common	40~60	0.05~0.1	1~5	1~5	10~50	30~50	5~10
Be poor	<40	<0.05	<1	<1	<10	<30	<5

RETRACTED

## Data Availability

The data used to support the findings of this study are available from the corresponding author upon request.
